# Study on the Application of Traditional Chinese Auspicious Images in Environmental Art Design Based on VR Senses

**DOI:** 10.1155/2022/1189613

**Published:** 2022-09-17

**Authors:** Zhou He

**Affiliations:** Cheng Nan Academy, Hunan First Normal University, Hunan Changsha 410000, China

## Abstract

Virtual reality is high-tech involving multiple disciplines developed at the end of the 20th century. Virtual reality technology can be used in many fields, such as remote control, business, education, entertainment, visual simulation, military, art, architecture, and network. Essentially, virtual reality technology has three basic characteristics: immersion, interaction, and imagination. This study analyzes the advantages of VR technology in the specific application of environmental art design based on case studies and considers the impact of VR technology on human beings from multiple dimensions such as sociology and philosophy. First, it analyzes the application and advantages of VR technology in various stages of the environmental art design. Secondly, combined with cases, it explains the advantages of VR technology in four directions: exhibition, interior, landscape, and planning. Then, it finds out the problems in the application and their solutions. In addition, to solve these problems, you need to explore the answers from more fields such as philosophy and sociology. Then, it discusses the development trend of environmental art design under VR technology and how designers should keep up with the time. Finally, as a designer of the new era, we apply VR technology to our own design and creation practice. We also analyzed the many forms of expression of auspicious images. Through the actual research and induction of modern designers, we summed up its main forms and expressions and drew some conclusions that everyone recognized, which can provide a reference for future designers.

## 1. Introduction

Chinese auspicious imagery is a unique landscape of oriental culture. It has a wide range of materials, rich and diverse content, and a long history, which cannot be replaced by other forms [1, 2]. The Chinese people use auspicious images to give them a peaceful environment with good wind and rain. Hope for a harmonious family, a happy life, and full children and grandchildren. These simple ideas and good wishes are transformed into auspicious and happy artistic shapes by people. People regard these pictures of auspicious themes as the great magic weapon for all souls, and they run through their clothing and residence, witchcraft beliefs, life etiquette, and many other folk activities [3].

The most commonly used is the comprehensive use of homophonic, metaphorical, and symbolic techniques. It is composed in a way that is suitable for understanding so that the form and content are combined ingeniously, which is pleasing to the eyes and ears [4]. These patterns can be said to be intentional in pictures and auspicious in meaning, have become popular among the people, and have even reached the level of common people and conventions. The application of traditional auspicious images in environmental art design is mainly manifested in brick carvings, stone carvings, wood carvings, calligraphy and paintings, furnishings, and other physical forms [5, 6]. People hope that through these entities endowed with auspicious images, they can place their trust in themselves and their families. At the same time as the good wishes of the collective and the guests, they come to beautify life and decorate the environment. While they respect the natural environment and function, homophony, meaning, and symbolism have become important forms that affect their environmental design [7].

Virtual reality (VR for short) technology, also known as spiritual technology, is high-tech involving multiple disciplines developed at the end of the 20th century. It integrates computer technology, sensing technology, simulation technology, and microelectronic technology [8, 9]. The ideal virtual reality technology is to use these technologies to create a virtual environment through the computer, through the functions of sight, hearing, touch, taste, smell, etc., so that the user can feel the same as in reality [10]. It will create an immersive feeling and enable direct user interaction with the environment. Virtual reality technology brings revolutionary changes in many disciplines such as artificial intelligence, CAD, graphic simulation, virtual communication, remote sensing, entertainment, and military simulation training, and will have far-reaching consequences for a country's national defense, military, politics, economy, culture, and even daily life [11]. There are three main characteristics of VR technology, and each of them is related to each other: (1) *Immersion*, which means that the user feels the real virtual world, so you can measure the immersion by looking at the immersion of the user into the virtual environment. (2) *Real-time interactivity*: Interactivity must first ensure the authenticity, effectiveness, and real-time nature of user operations, observe, and operate the simulated environment in a natural way, and get natural feedback. (3) *Rich ideation*: To get immersion, there is a necessary condition first, which is conception. In the virtual environment, a richer imagination is generated, which is realized through the immersion and real-time interaction it generates, and at the same time, the human cognitive limit is further broadened through the user's wide associative space.

The application of virtual reality technology is very wide, including remote control, business, education, entertainment, visual simulation, training, military, art, scientific visualization, criminal investigation, and network application [12, 13]. In the aspect of perfect e-commerce, the sales products are displayed in a three-dimensional form, and customers can have a more comprehensive understanding of their products by observing and operating them [14]. The probability of deciding to buy is greatly increased, bringing more sales opportunities and profit [15]. Virtual reality technology can use 3D courseware with interactive functions, and students can get a more profound experience through practical operation, which is conducive to the digestion and understanding of knowledge. The introduction of the three-dimensional method will definitely cause a new round of visual impact and increase the number of visits to web pages [16]. Through virtual reality technology, roles such as three-dimensional virtual hosts can be established on the site to attract visitors, thereby increasing the company's reputation.

Visual stimulation is an important field of virtual reality application, which has important uses in urban planning, environmental art design, architectural design, and so on [17]. Designing a virtual three-dimensional model according to the virtual reality scene to establish the entire virtual scene environment can fully display the real environment in front of us and make people feel a sense of reality similar to field observation. People can be placed in the scene and can see the planning effect from any angle and real-time interaction, and obtain an unprecedented intuitive feeling [18]. The virtual 3D model is easy to modify and can realize information management in the virtual environment, such as information query and analysis functions. Visual simulation provides a good solution for construction, urban planning, real estate, and other industries, which is an important application aspect [19].

Environmental art has a broad connotation, and in addition to including “artwork” designed to beautify the environment, it should also include “HappeningART,” “LandART,” and what the architectural world calls “art,” “Landscape Art (Landscape),” etc. [20]. The environmental art design can be divided into two aspects: material form and ideology. Material form mainly refers to the material elements that constitute the environmental landscape, and these material elements can be divided into different types according to different materials. Ideology mainly refers to the spiritual factors that influence and guide people's behavior, such as religious beliefs, folk customs, aesthetic concepts, social systems, ethics, and so on [21]. The relationship between the elements of environmental design is like the symbiotic chain of biological communities, which maintains the germination of all things in nature and is in a state of dynamic equilibrium [22]. This state is precisely the goal that modern environmental art design should pursue. Its task is to design an optimized “human-environment system,” which will show the coexistence of human beings and the environment and the balance between human beings and the environment at a new high level [23].

A long time ago, researchers used drawing tools to design the drawings of the architectural environment, and the design steps were very cumbersome, error-prone, long-term, and expensive [24]. Since the application of computers to the design industry, designers can use computer graphics software to draw drawings and then use 3D software (such as 3DMAX) to draw the virtual scene, render the picture from the best angle of the scene, and print it out as the rendering of the architectural environment. Through this mode, the work efficiency is greatly improved [25]; people seem to have an intuitive feeling of the real architectural environment from the design of the renderings. From the 1990s to the present, this method has become a popular design mode, which has been accepted by the majority of design companies, planning departments, decoration companies, garden departments, architectural design institutes, and other departments [26]. With the continuous improvement of scientific and technological levels, people find that no matter how detailed these designs are, no matter how exquisite the performance of renderings, they can never give people a very intuitive feeling [27]. At most, people only observe through the performance of renderings. The effect map is just a static map, which only expresses the main body of the whole environment, but cannot observe other details. Therefore, it is impossible to give an immersive feeling [28]. Through virtual reality (VR) technology, this problem can be solved very well. The entire environment must be modeled into a virtual scene through 3D software, and the models in the scene must be interactively controlled through VR technology. That is, people can observe the scene in a first-person way through computer input devices, such as mouse, keyboard, and joystick, and feel the same feeling as the real scene [29]and effects that cannot be achieved by ordinary methods. In addition, the model in the virtual scene is easy to modify, and other functions can be added on this basis, for example, the query function: you can operate the virtual scene through the computer input device to obtain some information in the computer scene; analysis function: through simple operations realize some engineering applications, such as measuring distance and obtaining position coordinates [30].

Due to the intuitiveness of the application of virtual technology, it breaks the communication barriers between professionals and non-professionals, enabling various departments to communicate through a unified simulation environment, and can find problems, reach consensus and solve some design problems more quickly [31]. In addition, the virtual design of the building environment can also be carried out through virtual technology. Before the construction is carried out, the virtual design scheme can be discussed with the customer, and through the modification of the scheme, the production and construction can be put into production until the customer achieves a satisfactory effect. In this way, a lot of capital and manpower investment can be saved, and it is a brand-new design concept and design method [32].

Our study has the following innovations. First, the previous research on VR technology in environmental art design is more focused on the research from the perspective of computer science, and it is more inclined to the production and development of software, while this paper focuses more on the arts and humanities. Secondly, it is necessary to integrate display, interior, landscape, planning, and design, and discuss the relationship with VR technology application from a comprehensive perspective. In addition, we have our own new understanding of environmental art design from the perspective of VR technology and discuss the design trends under VR technology. We first integrated exhibition, interior, landscape, planning, and design, and discussed the relationship with VR technology application from a comprehensive perspective. Finally, we also analyzed the actual meaning of Chinese traditional auspicious pattern.

## 2. Methods

This research mainly uses the currently relatively popular visual technology,. panorama, also known as panoramic virtual reality (also called virtual panorama). Both traditional 3D technology and network 3D technology represented by VRML use computer-generated images to build 3D models, while panorama technology uses real photos to build a virtual environment and follows the pattern of photo shooting, digitization, image stitching, and scene generation, a complete VR creation which makes panorama technology more simple and practical [33]. The advantages of panoramic technology are as follows: the method is simple, the design cycle is shortened, the development cost is low, the effect is still high, and the application is relatively wide, so it is more popular at present. Especially with the continuous development of network technology, its superiority has become more obvious. People can do 360 online, panoramic observation, and free browsing through interactive operations, so as to experience the three-dimensional VR visual world. In this case, the use of VR glasses can also produce a strong sense of immersion. It also has drawbacks: panoramic virtual reality, also known as photorealistic virtual reality displays [33]. It only offers viewer zoom in and out and 360. It allows browsing products in the same direction, but cannot provide deeper interaction, so it is not sufficient in terms of interactivity.

In the creative process, the main tools used are Ricoh THETA S panoramic camera, Google Cardboard glasses, tripods, telescopic poles, desktop computers, smartphones, etc. The Ricoh THETA S is a typical 360. Panoramic camera. Different from ordinary cameras, the panoramic camera has two fisheye lenses at the front and the rear, and the front and rear lenses of the camera will take a picture of about 180 degrees. The super wide-angle photo of the fuselage, and then through the internal calculation of the fuselage, the two photos are combined into one, and a panorama similar to the Boodle Street View will be generated [34]. The panoramic camera can record all the image information of the front, back, left, and right at one time, without artificial synthesis in the later stage, and no need for multilens stitching. Its principle is based on the principle of bionics using the spherical mirror transmission and reflection principle of physical optics to image the information of 360 degrees horizontally and 180 degrees vertically at one time, and then uses the software that comes with the hardware to convert, and present the picture in a way that the human eye is used to [34]. Ricoh THETA S was released in September 2015. With its small size, lightweight, and built-in WiFi function, users can easily transfer to smart devices and social networks to share with others after shooting (Figure 1).

A 360-degree panoramic camera has the following characteristics: (1) Overwhelming wide-angle camera. Panoramic camera level 360-degree 180-degree is shown in Figure 2. The panoramic camera subverts the concept of the previous wide-angle camera. For camera products, shooting has no dead ends. (2) The file size is small, the download is fast, and ordinary computers and smartphones can be browsed and viewed smoothly, without the need for a special workstation. There are no technical obstacles to network promotion. (3) The spherical curved image can be transformed into the usual semicurved view. The image captured by the fisheye camera can be converted into a normal plane view suitable for the human eye through the correction of the camera's internal software and the processing of surface expansion.

Google Cardboard glasses are cheap 3D glasses launched by Google at the 2015 Google I/0 developer conference held in San Francisco, USA, on May 29, 2015. The appearance is shown in Figure 3. As shown in the spectacle body 3, through the principle of lens and screen, the virtual image is presented at the distance of people's bright vision to achieve an immersive sense of virtual reality. At present, most domestic virtual reality glasses use this principle, but they have been carefully packaged, making it more comfortable to wear. The parts in the Google Cardboard carton include a paper plate, lenticular lens, magnet, rubber band, NFC sticker, and magic sticker. After a simple folding, a viewfinder and a slot for a smartphone can be formed. The semicircular groove is just enough to bury a person's face and nose. Although Google Glass looks like a relatively simple box glasses, this glasses can bring a VR experience with a smartphone. Moreover, it is lightweight, has no cable restrictions, and is more comfortable to wear, making it a good choice for experiencing panoramic VR.

Other hardware devices. Tripod: it fixes the panoramic camera to prevent lens shake; telescopic pole: it provides a position for the camera close to the height of the human eye; desktop computer: it renders renderings and uploads renderings to the cloud for panoramic synthesis; smartphone: it operates the panoramic camera and the RICOH THETA S app.

The third-party applications are as follows: (1) SketchUP: SketchUp is a very popular and simple 3D design software in the field of environmental art design, which is likened to the “pencil” in electronic design; (2) 3ds Max: it is a 3D animation rendering and production software based on PC system developed by Autodesk, and its predecessor is 3DStudio series software based on DOS operating system; (3) V-Ray renderer: V-Ray for 3ds Max is a third-party renderer for 3ds Max, designed and produced by Chaos Software, a professional rendering engine company, with ray tracing and global illumination renderers; (4) Dsketch: it is a third-party plug-in of SketchUp, providing VR scrutiny function; (5) Ricoh Jingda S: it is an application system based on a smartphone, which provides the function of viewing panoramic photos in VR [35].

The desktop VR experience mainly uses the computer to display the screen, uses the mouse, or manipulates the objects in the scene. Therefore, in this case, as an auxiliary experience, it is mainly used when the number of participants is large, such as communication plans and presentations.

Immersive VR experience is the main way of experience in this case, because it is highly perceptible, lightweight, and portable [35]. You can complete the VR experience by simply inserting the smartphone into the card slot, and it can be used at all stages. In the design preparation stage, the author watched the scene map through the immersive VR experience; in the design deliberation stage, the immersive experience can better experience the sense of the scale of the design in the “first-person” way in the scene; in the design display stage, the owner also uses the immersive experience feels the design effect.

## 3. Result and Discussion

### 3.1. Site Surveying and Mapping Stage

The purpose of applying VR technology in the lobby design stage is to allow the author to be immersed in the VR panoramic construction site “anytime, anywhere” without being limited by time and space, so that the characteristics and specific situation, so as to make a design that is closer to the actual situation. In the process of designing the lobby, we used Ricoh THETA S for panorama shooting in addition to regular photos. First, place the Ricoh THETA S on a tripod, and try to place the camera in the middle of the environment you want to shoot to ensure that you can shoot in all directions of the space. Then, turn on the camera and enable Wi-Fi to connect the smartphone to the Wi-Fi to control the camera [36]. In order not to appear in the picture of the author's own image, use a smartphone to control the camera through Wi-Fi to shoot, and the picture will be automatically saved after shooting.

As shown in Figure 4, it is a panoramic photo taken before the renovation of the sloping roof and the south courtyard. After shooting, the spherical image can be converted into a normal plane view (i.e., standard view). The image captured by the fisheye camera is corrected by the camera's internal software, and the image is expanded to convert it into a normal plane view suitable for the human eye. Just zoom with your finger to get viewing in all directions. The standard view is for desktop VR experiences. If you want to use VR glasses for an immersive experience, you need to adjust the “standard screen” mode to “VR view (dual lens),” which is the VR mode. The dual lens can better simulate the observation range of two eyes. With VR glasses, there will be an immersive experience.

In addition, we also used Ricoh THETA S to take a panoramic camera in some spaces, which can better restore the scene of the lobby, especially for a larger space. A panoramic picture cannot restore all the details, but a panoramic video can solve the problem. In the later stage, the corresponding software is also used for decoding to achieve the effect of VR viewing. However, the resolution of the panoramic video is slightly lower (Figure 5).

The panoramic shooting of the site, even if the person is not on-site, the Ricoh Jingda APP in the smartphone can watch the panorama of the construction site, cooperate with Google Cardboard glasses for immersive VR roaming, or output the panorama to the computer for desktop VR roaming, suitable for discussion and communication with owners.

After the author's practice test, the use of virtual panorama observation can indeed more intuitively and comprehensively grasp the state of the scene. Compared with ordinary photos, it is like stitching photos from each angle in sequence, restoring the whole scene of the scene. In the process of summarizing the surveying and mapping data and drawing CAD, it can also better assist the drawing of CAD. In addition, the immersive experience enhances the feeling of the atmosphere of the whole space, and then bursts out unexpected design inspiration.

### 3.2. Design Deliberation Stage

In the design deliberation stage, it is even more necessary to proceed from a practical point of view, starting from the needs of space users to grasp the scale, material, and style of the design. Through VR deliberation, the owner can also participate in it, so as to make more targeted, design works that are more in line with the needs of users in this environment.

In the design deliberation stage, the author mainly used a SketchUp VR plug-in Dsketch developed by Beijing Lefang Technology Co., Ltd., which can effectively assist in deliberating the rationality of the spatial scale. In the process of design deliberation, using this plug-in, it seems to be immersed in the draft space of 3D modeling, getting an immersive space effect and experiencing the sense of scale of the design more accurately. The specific steps for using the Dsketch plug-in for design deliberation are as follows. First, the Dsketch plug-in needs to be installed and user registration is done. Pour the modeled model into SketchUp, and set a camera viewpoint close to the height of the normal person's field of view. In the second process, the camera set in SketchUp simulates the function of a panoramic camera and shoots the scene 360 degrees. Then select Dsketch in the expansion project, click “Generate Panorama,” and “Copy Path,” “Click Upload to Mobile Phone,” a QR code will be automatically generated on the computer. Scan the QR code with a mobile device, and the generated VR panorama will be transmitted to the mobile terminal. Click the VR mode, put the mobile device into the VR glasses, and you can watch in VR. With the rotation of the body, the VR field of vision is also constantly changing, and you can experience the sense of spatial scale from each angle, and provide effective feedback on the design. This plug-in is specially used for SketchUp software, and SketchUp is a good design review software for indoor and outdoor design, so the Dsketch plug-in can be applied to the review of many aspects of Huanyi design. The effect is more direct, the tools are easier to obtain, and the operation is more convenient.

Using the Dsketch plug-in for VR deliberation first makes up for the author's lack of spatial imagination and spatial scale control. After wearing VR glasses, it is like entering the courtyard under deliberation, and can design and conceive more intuitively and more freely. Secondly, “immersive” design deliberation can better discover the deficiencies in the design, and also generate unexpected inspirations and realize the expansion of thinking; furthermore, and the most important point, the VR deliberation scene can be viewed through a smartphone. Send it to the owner, so that the owner can check the design and put forward opinions during the design process, which realizes the good communication of the design, and makes the design fully reflect the wishes of the users of the environment.

Combined with the owner's own characteristics, let VR technology bring beautiful, interactive, and easy-to-operate display methods, and shorten the distance between the performance effect and the owner, so that the design ideas can be understood and expressed as much as possible, and the design scheme is also to have humane care.

In this case, the performance of the outdoor effect is mainly drawn with the SketchUp software, so it is necessary to create a panoramic view of the effect map. This requires certain settings in the render plug-in V-Ray Camera. When the model is completed, the material mapping is carried out according to the conventional method, and the setting parameters of the V-Ray camera need to be changed. After positioning the camera according to the requirements in the scene, you need to change the camera type in the V-Ray panel from “Standard” to “Spherical,” check “View Override,” and select “360 Degrees.” Then, set the image aspect ratio in the output column to 2 : 1, and set the desired output image size.

After completing the above two steps, click the render button to render, and when the rendering is over, the rendering of the 2 : 1 ratio is completed (Figure 6(a)). After this step, it is necessary to perform panoramic synthesis on the renderings, which can be synthesized by using the Pano2VR software, but this method is more complicated and time-consuming. Moreover, online panorama synthesis can greatly save time and effort. Log in to https://www.justeasy.cn to upload the renderings directly. The system will automatically synthesize a virtual panorama and generate a QR code to scan it to view the panorama. Select the VR mode and use VR glasses to perform VR roaming (Figure 6(b)). At the same time, the drawings can be uploaded, and the drawings can be viewed while watching the VR roaming, which greatly meets the needs of nonprofessional customers. The rendered VR panorama effect is more realistic, adding a certain interest and freshness.

The performance of indoor effects is mainly produced by 3ds Max software and *V*-Ray rendering. Therefore, 3ds Max and VR are combined to perform VR processing on renderings. Compared with ordinary renderings, some related parameter settings need to be changed during rendering. After the materials and lights have been assigned, first adjust the camera type in the V-Ray panel from “Standard” to “Spherical,” check “View Override,” and select “360 Degrees.” Then, set the aspect ratio of the image in the output column to 2 : 1, and set the image size of the rendering output. In order to ensure the VR effect, it is generally set to 5000 × 2500.

In addition, it is necessary to add a target camera to the scene and ensure that the camera can capture the space and objects to be presented within a 360-degree range. After the camera is set up, the renderings are rendered. After a few hours, a rendering with a ratio of 2 : 1 will be generated (Figure 7), and it will be integrated into the online cloud to synthesize the panoramic VR renderings (Figure 8). Select the VR mode and cooperate with VR glasses to get an immersive VR experience (Figure 9). In addition, the interactive functions are enriched by combining elements such as CAD drawings, design instructions, and background music (Figure 10).

The panoramic VR method is used to intuitively express the effect of the design, especially combined with CAD drawings, and has a certain interactive function, which makes the display of information more abundant. In addition, the shareability and ease of dissemination of the network-based panoramic VR in this case is very suitable for the age group of the owner, which shortens the distance between the design and the user.

### 3.3. The Practical Significance of Auspicious Patterns

The design language of the lobby is mainly reflected in that the traditional structural form is used in the structural space, the sloping roof is adopted, and the wooden beam frame is maintained. In the treatment of the wall, the water splashes, representing the Yellow River culture and the wishful patterns representing the auspicious patterns are skillfully grafted, and expressed in the form of reliefs, which not only reflects the regional culture, expresses the meaning of the auspicious patterns, but also increases the level of the space. The traditional furniture used in the interior has been simplified and reformed, and it is more modern on the premise of maintaining the original charm. The selection of accessories is also reflected in the combination of screens and paintings, and the content of the paintings is based on local characteristics (Figure 10).

The conference room is located on the north side of the lobby on the first floor, only on the first floor, so the roof adopts a sloping roof, and the roof structure adopts a traditional herringbone beam frame. The beam frame that is too large makes the space bulky, so the beam frame is refined, but the load bearing is considered. Therefore, the number of beam frames is increased to form a sequence, and the organic combination of lighting fixtures and beam frame structures can be called beautiful. Due to the small space, the color tone of the wall is relatively uniform and there are few changes, in order to pursue the integrity of the space. The combination of folding screen and Chinese painting is a favorable example. It breaks the rigidity of the space and reflects the regional characteristics of the space.

The clubhouse suite is located on the south side of the second floor, with a good line of sight and unobstructed outdoor scenery. As the entrance of the suite and the distribution center of the evacuation space, a small front hall is designed in front of the living room to evacuate the crowd and ensure that the people in the living room are not disturbed, so that the area of the living room will be reduced. The top of the living room is treated as a flat top, making its aspect ratio more intimate. In order to reflect the publicity and transparency of the living room, in the living room only door covers are designed for the entrance and exit. The transparent window uses auspicious clouds as the pattern, the painting uses the “lotus” as the material, and the poems are used to extend the artistic conception of the picture (Figure 11).

The top surface of the bedroom also adopts the plane treatment method to ensure the intimacy of the space. The main and secondary treatment of the façade is distinct. The main wall of the seat back is made of wood to soften the space interface. The pineapple lattice wood in the middle can not only reflect the tradition, but also promote the unity and connection with other spaces. The jade pendant as a pendant reflects the grade of space. The design of the table lamp is extremely refined, and there is not a little too much language. The ingenious combination of pillow shape and traditional Fang Sheng parquet not only reflects beauty but also contains profound meaning. The bed flag of red satin jacquard on the bed can further deepen the festive atmosphere.

The study room is a smaller space in the suite, and it just adds a little space for reverie while satisfying reading and office work. The bookcase adopts the form of a wooden duo bao pavilion, which can not only achieve the connection with other spaces, but not lose traditional cultural symbols, but also better meet the functions. The office furniture has been refined and summarized in design, and the lower volume of Chinese classical furniture is skillfully combined with the desk of modern panel furniture, which not only reflects the classical beauty of traditional furniture but also has a modern sense. Because the space is small, the choice of accessories is relatively simple, but on the opposite wall is a meticulous painting by Li Qingzhao, a representative of our Jinan literati, a poet of the graceful school, which is intended to strengthen the regionality of the space and play the finishing touch.

## 4. Conclusions

VR and other technologies have penetrated into the field of environmental art design, are changing the means of modern design, and its application will be more in-depth. With the continuous development of VR technology, the application methods in environmental art design will be more abundant, and it will also bring endless creative inspiration to designers.

In our study, we do some analysis on the application of VR technology in various stages of environmental art design, and based on the different characteristics of exhibition design, interior design, landscape design, and planning design, combined with specific cases, it can be concluded that the application of VR technology is more specific. Research and analysis. We also found that there are some problems in the practical application of VR technology, such as the decline of the designer's own ability caused by VR technology, the excessive pursuit of technology and neglect of content in design, and the insufficient “humanization” of VR experience. In my own practice, I try to avoid these problems, not using VR technology as a design gimmick, but as a means to make design more humane, using VR technology to assist the author to better stand in the perspective of environmental users' question.

Finally, we combined with actual cases to explain the application of traditional Chinese auspicious images in environmental art design. Through the form of space, the architectural structure analyzes the characteristics of Chinese style space and how to use the architectural structure to design the interior space in the design. The second is to create a comfortable, easy-to-use, and meaningful interior space through the combination of the facade form and traditional auspicious symbols. The last is to enhance the cultural atmosphere of the space through the design and placement of accessories.

In the research, no higher-level VR technology is involved, so the VR experience is still at a relatively elementary stage. Moreover, the application method is relatively simple, and multiple VR technologies are not used to participate in the design, which makes the experience of the project need to be improved. The limitations of panoramic technology have resulted in not fully volatilizing all the advantages of VR technology, especially the interactive sense of VR technology has not been fully reflected. In the design creation, no matter what kind of technology is used, the purpose is to make a “humanized” design. Because in the final analysis of the design of environmental art, people exist as the subject of use. The user is the starting point and the destination point of the design. Therefore, looking forward to the future, the application of VR technology in environmental art design must always revolve around the physical and psychological needs of environmental occupants and users, and humanistic care needs to be fully reflected in all stages of application. The full release and satisfaction of “humanization” should be the pursuit of applying VR technology to environmental art design.

## Figures and Tables

**Figure 1:** Ricoh THETA S top view detail (a) and hardware diagram of the fisheye lens (b).

**Figure 2:** Panoramic camera (a) and monocular viewing (b) angle comparison.

**Figure 3:** Google cardboard glasses (a) and how google cardboard works (b).

**Figure 4:** Lobby spherical image, flat view, and VR view (dual camera) mode.

**Figure 5:** VR panoramic video.

**Figure 6:** Rendered 2 : 1 ratio renderings (a) and VR viewing after compositing the scene (b).

**Figure 7:** 2 : 1 aspect ratio rendering renderings.

**Figure 8:** The generated panorama rendering can be used for desktop VR experience.

**Figure 9:** Panorama in VR mode with VR glasses for immersive VR experience.

**Figure 10:** Exhibition hall renderings.

**Figure 11:** Suite living room design.

## Data Availability

The experimental data used to support the findings of this study are available from the corresponding author upon request.
